The article "Effect of MiR-375 Regulates YAP1 on the Invasion, Apoptosis, and Epithelial-Mesenchymal Transition of Cervical Cancer HeLa Cells" was retracted in 2023. Reasons: signs of a paper mill; compromised peer review; unreliable results or conclusions.

# Effect of MiR-375 Regulates YAP1 on the Invasion, Apoptosis, and Epithelial-Mesenchymal Transition of Cervical Cancer HeLa Cells

**DOI:** 10.1155/2021/3088723

**Published:** 2021-09-01

**Authors:** Yi Hu, Yan Ma, Guifang Luo, Wenyan Liao, Shufen Zhang, Genlin Li

**Affiliations:** The First Affiliated Hospital, Department of Obstetrics and Gynaecology, Hengyang Medical School, University of South China, Hengyang, Hunan 421001, China

## Abstract

Yes-associated protein 1 (YAP1) is an important signaling pathway activator molecule. Studies have shown that it is involved in the occurrence of malignant tumors. This study identified a microRNA (miR/miRNA) targeting the 3′ untranslated region (3″ utr) of the YAP1 gene and evaluated its biological impact on human cervical cancer cells and related molecular mechanisms. qPCR and western blotting were used to detect the levels of miR-375 and YAP1 in HeLa cells. TargetScan software was used to identify the binding sites of YAP1 and miR-375. The MTT method was used to determine the viability of HeLa cells transfected with miR-375 mimic and YAP1 interference vector, the Transwell chamber experiment was used to detect the invasion of HeLa cells after transfection, the apoptosis of HeLa cells after transfection was detected by flow cytometry, and the western blotting was used to detect the epithelial mesenchymal transition (EMT) of HeLa cells after transfection. The expression of miR-375 in HeLa cells was significantly lower than that of normal control cervical cells, and the expression of YAP1 in HeLa cells was significantly higher than that of normal control cervical cells. TargetScan analysis showed that miR-375 was bound to the 3′ UTR of YAP1. qPCR and western blot analysis showed that transfection of miR-375 mimics inhibited YAP1 expression in HeLa cells. Transfection of miR-375 mimic and YAP1 interference vector inhibited HeLa cell invasion and EMT and promoted HeLa cell apoptosis. These findings indicate that miR-375 inhibits the malignant development of human cervical cancer cells by regulating the expression of YAP1.

## 1. Introduction

Cervical cancer is one of the most common malignant tumors in gynecology. It has a high morbidity and mortality rate, and it is showing a young trend. As women's labor participation rate increases and life expectancy increases, it is of great significance to improve women's health and quality of life [1]. The occurrence of cervical cancer is a process of multifactor influence and multistage development, and its regulatory mechanism is complex. Studies have shown that epigenetics plays an important role in the occurrence and development of tumors [2]. MicroRNA (microRNA, miRNA) is abnormally expressed in a variety of malignant tumors and participates in the occurrence and metastasis of malignant tumors. MiRNAs with abnormally elevated expression accelerate tumorigenesis by inhibiting tumor suppressor factors, and miRNAs with reduced expression inhibit tumorigenesis by negatively regulating the expression of oncogenes [3, 4]. miR-375 has been confirmed to be related to the occurrence of cervical cancer. The serum level of miR-375 in patients with cervical cancer has decreased significantly, and it has a similar effect to tumor suppressor genes [5], but its specific mechanism of action has not yet been elucidated. Yes-associated protein 1 (Yes-associated protein 1, YAP1) is an important signaling pathway activation molecule. The abnormal increase of YAP1 expression leads to the continuous proliferation of downstream tumor cells, which participate in the early occurrence of malignant tumors [6]. Epithelial-mesenchymal transition (EMT) is the process by which epithelial cells transform into mesenchymal cells. It is a common physiological phenomenon in mammalian development. However, abnormal EMT will cause epithelial cancer cells to migrate and invade and participate in malignant evolution of tumors. At present, the mechanism of how cervical cancer cells invade surrounding cells is not clear, but it is generally believed that EMT plays an important role in this process [7].

Therefore, this study used cell proliferation, invasion, and apoptosis experiments to study the effects of miR-375 and YAP1 expression on the proliferation, invasion, apoptosis, and EMT process of cervical cancer cell line HeLa, aiming to provide data for the clinical diagnosis and treatment of cervical cancer stand by. The specific research is as follows.

## 2. Materials and Methods

### 2.1. Experimental Materials and Reagents

Normal cervical epithelial cells H8 and cervical cancer cells HeLa were purchased from the Shanghai Cell Bank; the RPMI 1640 culture medium and fetal bovine serum (FBS) were purchased from GIBCO, USA; the primers of miR-NC, miR-375 mimic, si-NC, si-YAP1, miR-375, and U6 were all purchased from Shanghai Gima Co., Ltd.; wild-type (WT) and mutant (MUT) YAP1 plasmids were synthesized by Shanghai Shenggong Biological Company; the RT-PCR kit, YAP1, *E*-cadherin, *β*-catenin, vimentin primary antibody and the corresponding secondary antibody, and Transwell chamber were all purchased from Sigma in the United States; RNA extraction kits, Lipofectamine^TM^ 2000, MTT, and apoptosis kits were all purchased from Wuhan Boster Biotech; both Trizol reagent and the luciferase detection kit were purchased from BioVision, USA.

### 2.2. Cell Culture and Transfection

H8 and HeLa cells were cultured in the RPMI 1640 medium containing 10% FBS, 100 *μ*g/ml streptomycin, 2 mmol/L glutamine and 100 U/ml penicillin at 37°C, and 5% CO_2_. When the cells grew to 70–80% confluency, the transfection followed the Lipofectamine ^TM^ 2000 operating instructions to combine miR-375 mimic (miR-375 mimic) and negative control (miR-NC), and YAP1 interference vector (si- YAP1) and negative control (si-NC) were, respectively, transfected into HeLa cells and continued to be cultured.

### 2.3. PCR Detection

Untreated H8 and HeLa cells and cells transfected according to the abovementioned operation were collected and centrifuged at 4°C and 8 cm 1000 r/min for 10 minutes, and the supernatant was discarded. The Trizol method was used to extract total RNA from cells, taking 1 *μ*g of total RNA and performing reverse transcription according to the instructions of the reverse transcription kit. Fluorescent real-time quantitative PCR was used to detect the expression of miR-375, 95°C for 3 minutes and then 95°C for 10 seconds., 60°C for 15 s, 72°C for 1 min, a total of 40 cycles. U6 was used as an internal reference, and related primers are shown in Table 1. The quantitative results were analyzed using the equation 2^−ΔΔ^CT^^ method; Δ*Ct*(*n*)=*Ct* target gene (*n*)−*Ct* internal reference gene (*n*); ΔΔCT(*n*)=Δ*Ct*(*n*) − Δ*Ct*(1).

### 2.4. Western Blot Detection

Untreated H8, HeLa cells, and transfected cells of each group were collected and centrifuged at 4°C and 8 cm 1000 r/min for 10 min, and the supernatant was discarded. They were operated on ice, added with 50 *μ*L of RIPA lysate, and centrifuged at 4°C and 12000 g for 15 min, and after 30 min, the supernatant was taken for BCA protein quantification. 40 *μ*g of sample was added to the buffer solution, boiled at 100°C for 5 minutes, and separated by 12% polyacrylamide gel electrophoresis (SDS-PAGE), polyvinylidene fluoride (PVDF) was transferred to the membrane, and TBST solution was blocked for 2 hours. Primary antibodies YAP1 (1 : 1000), *E*-cadherin (1 : 1000), *β*-catenin (1 : 1000), vimentin (1 : 1000), and GAPDH (1 : 1000) were added and incubated overnight at 4°C. The next day, horseradish peroxidase- (HRP-) labeled rabbit anti-mouse secondary antibody was added and incubated at room temperature for 1 hour for color development. Using GAPDH as an internal reference, Quantity One software analyzed the gray value of the band, and the ratio of YAP1, *E*-cadherin, *β*-catenin, Vimentin, and GAPDH gray value was used as the relative expression of YAP1, *E*-cadherin, *β*-catenin, and vimentin. The experiment was repeated three times.

### 2.5. MTT Experiment

Each group of HeLa cells in the logarithmic growth phase was taken and trypsinized to prepare a single cell suspension, and the cell concentration was adjusted to 3 × 10^4^ cells/mL. 200 *μ*L of cell suspension was inoculated into a 96-well plate and placed in a 37°C, 5% CO_2_ incubator for 24 h, 48 h, and 72 h, 20 *μ*L of MTT solution was added 4 h before the corresponding time point, and the culture was continued for 4 h. 150 *μ*L of cells were added to each well and mixed well, and the absorbance (OD) was measured by using a microplate reader (490 nm). The experiment was repeated three times.

### 2.6. Transwell Chamber Experiment

Before the experiment, Matrigel glue was spread on the upper chamber of the Transwell chamber. Each group of HeLa cells in the logarithmic growth phase was taken and trypsinized to prepare a single cell suspension, and the cell concentration was adjusted to 8 × 10^3^ cells/mL. 200 *μ*L of cell suspension was inoculated in the upper chamber, and the medium containing 10% fetal bovine serum was added to the lower chamber of the Transwell chamber and cultured in a 7°C, 5% CO_2_ incubator for 48 hours. After taking out the chamber, the cells at the bottom of the upper chamber were scraped off, fixed with 4% formaldehyde, stained with 0.5% crystal violet, and washed with 95% ethanol. Five fields were randomly selected to observe the number of cell invasions under a microscope, and the results were averaged. The experiment was repeated three times.

### 2.7. Flow Cytometry

HeLa cells in each group in the logarithmic growth phase were taken, trypsinized, and centrifuged at 4°C and 8 cm 1000 r/min for 10 min. The supernatant was discarded, and the cells were resuspended. 20 *μ*L binding buffer solution was added and mixed, Annexin-V and PI were added, 400 *μ*L binding buffer was added, and the apoptosis of each group was detected by flow cytometry. The results were expressed as healthy living cells in the lower left quadrant (*Q*3) of the scatter diagram, the lower right quadrant (*Q*4) as early apoptotic cells, and the upper right quadrant (*Q*2) as necrotic and late apoptotic cells. Apoptosis rate = *Q*4 percentage + *Q*2 percentage. The experiment was repeated three times.

### 2.8. Luciferase Experiment

The bioinformatics software (http://starbase.sysu.edu.cn/) predicted the binding site of miR-375 and YAP1. The pGL3-YAP1-WT wild-type luciferase reporter vector containing the YAP1 3′UTR binding site was constructed, and the pGL3-YAP1-MUT mutant luciferase reporter vector without the YAP1 3′UTR binding site was constructed. The pGL3-YAP1-WT and pGL3-YAP1-MUT were cotransfected with miR-375 mimic and miR-NC into HeLa cells. After 24 hours, the medium was removed and the luciferase activity was detected. The calculation formula is relative fluorescence value = firefly luciferase fluorescence value/*Renilla* luciferase fluorescence value.

### 2.9. Statistical Methods

SDS1.4 software was used to calculate the sample CT value. The SPSS 22.0 software was used for processing, and the counting data are expressed by rate (%), and the *χ*^2^ test was used. Measurement data were expressed as mean ± standard deviation ($\bar{x}$ ± *s*), and the *t*-test was used for pairwise comparison between groups. The test level was *α* = 0.05, and *P* < 0.05 indicates that the difference was statistically significant.

## 3. Results and Discussion

### 3.1. The Expression of miR-375 and YAP1 in Normal Cervical Epithelial Cells H8 and Cervical Cancer Cell HeLa

The results showed that the expressions of miR-375 and YAP1 in H8 cells were 1.00 ± 0.08 and 0.46 ± 0.03, respectively, and the expressions of miR-375 and YAP1 in HeLa cells were 0.58 ± 0.04 and 1.09 ± 0.09, respectively. Compared with H8 cells, the expression of miR-375 in HeLa cells decreased, and the expression of YAP1 increased, and the difference was statistically significant (*P* < 0.05), as shown in Figures 1(a) and 1(b).

### 3.2. The Expression of miR-375 and YAP1 in HeLa Cells after Transfection of miR-375 Mimic and si-YAP1

The results showed that, after transfection of miR-375 mimic and si-YAP1, the expression of miR-375 in miR-NC, miR-375 mimic, si-NC, and si-YAP1 groups was 1.01 ± 0.08, 2.65 ± 0.24, 0.98 ± 0.08, and 1.02 ± 0.09, respectively, and the YAP1 expression was 1.23 ± 0.11, 0.74 ± 0.06, 1.28 ± 0.10, and 0.67 ± 0.05, respectively. Compared with the miR-NC group, the expression of miR-375 increased and the expression of YAP1 decreased in the miR-375 mimic group, and the difference was statistically significant (*P* < 0.05). Compared with the si-NC group, there was no change in the expression of miR-375 in the si-YAP1 group, and the expression of YAP1 decreased, and the difference was statistically significant (*P* < 0.05), as shown in Figures 2(a) and 2(b).

### 3.3. MiR-375 Targets the Expression of YAP1

The results showed that the bioinformatics software predicted that miR-375 and YAP1 had binding sites (Figure 3(a)). Luciferase experiment found that, after YAP1-WT and miR-375 mimic cotransfected HeLa cells, the cell luciferase activity decreased, and the difference was statistically significant (*P* < 0.05). But, after YAP1-MUT and miR-375 mimic cotransfected BGC-823 cells, there was no change in luciferase activity, and the difference was not statistically significant (*P* < 0.05). It shows that YAP1 is the target gene of miR-375, as shown in Figures 3(a) and 3(b).

### 3.4. MiR-375 Regulates the Effect of YAP1 on the Proliferation of HeLa Cells

The results of the MTT experiment showed that compared with the miR-NC group, the cell viability of the miR-375 mimic group decreased at 24 h, 48 h, and 72 h, and the difference was statistically significant (*P* < 0.05). Compared with the si-NC group, the cell viability of the si-YAP1 group decreased at 24 h, 48 h, and 72 h, and the difference was statistically significant (*P* < 0.05), as shown in Figure 4.

### 3.5. MiR-375 Regulates the Effect of YAP1 on the Invasion of HeLa Cells

The results showed that the cell invasion numbers of the miR-NC group and miR-375 mimic group were 132.64 ± 10.75 and 36.24 ± 5.66, respectively. Compared with the miR-NC group, the number of cell invasions in the miR-375 mimic group decreased, and the difference was statistically significant (*P* < 0.05). The number of cell invasions in the si-NC group and si-YAP1 group was 146.21 ± 13.29 and 30.07 ± 4.82, respectively. Compared with the si-NC group, the number of cell invasions in the si-YAP1 group decreased, and the difference was statistically significant (*P* < 0.05), as shown in Figures 5(a) and 5(b).

### 3.6. MiR-375 Regulates the Effect of YAP1 on HeLa Cell Apoptosis

The results of flow cytometry showed that the apoptosis rates of the miR-NC group and miR-375 mimic cells were 15.41 ± 2.02% and 43.65 ± 5.21%, respectively. Compared with the miR-NC group, the apoptosis rate of the miR-375 mimic group increased, and the difference was statistically significant (*P* < 0.05). The apoptosis rate of the si-NC group and si-YAP1 group was 14.78 ± 1.95% and 49.44 ± 5.73%, respectively. Compared with the si-NC group, the apoptosis rate of the si-YAP1 group increased, and the difference was statistically significant (*P* < 0.05), as shown in Figures 6(a) and 6(b).

### 3.7. The Effect of miR-375-Regulating YAP1 on the Expression of EMT-Related Functional Proteins

The results showed that compared with the miR-NC group, the E-cadherin and *β*-catenin protein content in the miR-375 mimic group increased and the vimentin decreased, and the difference was statistically significant (*P* < 0.05). Compared with the si-NC group, the *E*-cadherin and *β*-catenin protein content in the si-YAP1 group increased and the vimentin decreased, and the difference was statistically significant (*P* < 0.05), as shown in Figures 7(a) and 7(b).

## 4. Discussion

The current prevention and treatment strategies for cervical cancer only include vaccine prevention, surgery, radiotherapy, chemotherapy, RNA interference therapy, and hormone therapy. Although the cure rate of cervical cancer can reach 80%–90%, its recurrence rate is high, and the local control rate is poor, resulting in a decrease in patient survival rate [8]. Therefore, it is of great significance to find a safe and effective treatment method to improve the prognosis of cervical cancer patients and increase the survival time after surgery.

MiRNA consists of approximately 19–25 nucleotides and can be combined with the 3′-untranslated region- (3′-UTR-) specific binding site of one or more downstream target gene mRNAs to regulate the gene's transcriptional level. The expression is involved in multiple physiological and pathological processes such as cell differentiation, proliferation, and apoptosis. Abnormal expression of miRNA causes abnormal transcription and expression of its target genes, which provides important conditions for the occurrence and metastasis of malignant tumors [9]. With the continuous development of molecular biology technology in recent years, studies have found that a variety of miRNAs are abnormally expressed in cervical cancer [10], breast cancer [11], bladder cancer [12], and other malignant tumors, making miRNAs become new targets for targeted therapy of malignant tumors.

MiR-375 is involved in the pathological process of malignant tumors, and most scholars believe that it plays the role of tumor suppressor genes [13]. For example, in liver cancer, the expression of miR-375 is significantly reduced. After upregulating the expression of miR-375, it can target the expression of ErbB2 to induce liver cancer cells to stay in the G1 phase of the cell cycle and accelerate the apoptosis of cancer cells [14]. In gastric cancer, compared with normal gastric tissue, the expression of miR-375 in gastric cancer tissue is downregulated, and after the miR-375 mimic is transfected to achieve its overexpression, the migration and invasion of cancer cells are significantly inhibited [15]. In addition, miR-375 can also inhibit the proliferation of colorectal cancer cells, and its mechanism may be related to the targeted regulation of SP1 expression [16]. The results of this study showed that the expression of miR-375 in cervical cancer cells HeLa decreased, and after miR-375 mimic was transfected, the expression of miR-375 in HeLa cells increased, and the proliferation ability at 24 h, 48 h, and 72 h decreased significantly. Transwell experiment found that miR-375 can inhibit HeLa cell invasion, and flow cytometry detected cell apoptosis and found that miR-375 can promote HeLa cell apoptosis. The abovementioned results all indicate that miR-375 has a tumor suppressor effect, can inhibit the malignant behavioral activities of cervical cancer cells, promote their apoptosis, and can be used as a specific target for targeted therapy of cervical cancer.

YAP1 is the main effector molecule in the signal pathway Hippo-YAP, which plays an important role in regulating cell proliferation, invasion, apoptosis, and malignant transformation. Studies have shown that YAP1 is highly expressed in malignant tumors such as gastric cancer [4], laryngeal cancer [17], and triple negative breast cancer [18]. The results of this study showed that the expression of YAP1 in cervical cancer cells HeLa increased. After interfering with its expression, the proliferation and invasion of HeLa cells were inhibited, and the apoptosis rate increased. In addition, bioinformatics software found that miR-375 and YAP1 have specific binding sites, and luciferase experiments further proved that miR-375 can target and regulate YAP1 expression.

EMT refers to the transformation process from static, polar epithelial cells to active, nonpolar mesenchymal cells when cells are stimulated by the outside world. This process significantly increases cell migration, invasiveness, and resistance to apoptosis [19]. E-cadherin is an adhesion molecule, which is of great significance for maintaining the normal morphology and complete structure of epithelial cells. When its expression decreases, it will accelerate the metastasis of tumor cells [20]; *β*-catenin and *E*-cadherin play a synergistic role and are highly expressed in noninvasive or normal cells [21]; vimentin is an intermediate fibrous protein. The high expression of vimentin protein makes tumor cells more aggressive, and its increased expression in tumor cells is a sign of the occurrence of EMT [22]. The results of this study found that, after upregulation of miR-375 or interference with YAP1 expression, the protein content of *E*-cadherin and *β*-catenin increased and vimentin decreased. It shows that the high expression of miR-375 and the low expression of YAP1 can significantly inhibit the cell EMT process, reduce the proliferation and invasion of cancer cells, and promote apoptosis.

## 5. Conclusions

In summary, the expression of miR-375 decreased in cervical cancer cells, and the expression of YAP1 increased. After upregulating the expression of miR-375, the proliferation and invasion ability of cervical cancer cells decreased, the apoptosis rate increased, and the EMT process was inhibited. This may be related to miR-375-targeted inhibition of YAP1 expression. This study can provide data support for the clinical diagnosis and treatment of cervical cancer. In follow-up experiments, more genes related to cervical cancer can be explored, and new molecular targets can be provided for the targeted therapy of cervical cancer.

## Figures and Tables

**Figure 1:** The expression of miR-375 and YAP1 in H8 and HeLa cells. (a) The expression of miR-375 in H8 and HeLa cells; (b) the expression of YAP1 protein in H8 and HeLa cells; ^*∗*^*P* < 0.05, compared with the H8 group.

**Figure 2:** The expression of miR-375 and YAP1 in HeLa cells of each group after transfection. (a) MiR-375 expression in HeLa cells of each group after transfection; (b) YAP1 protein expression in HeLa cells of each group after transfection; ^*∗*^*P* < 0.05, compared with the miR-NC group; ^#^*P* < 0.05, compared with the si-NC group.

**Figure 3:** MiR-375 targets the expression of YAP1. (a) The binding site of miR-375 and YAP1; (b) luciferase experiment verifies the targeting relationship between miR-375 and YAP1; ^*∗*^*P* < 0.05, compared with the miR-NC group.

**Figure 4:** MiR-375 regulates the effect of YAP1 on the proliferation of HeLa cells. ^*∗*^*P* < 0.05, compared with the miR-NC group; ^#^*P* < 0.05, compared with the si-NC group.

**Figure 5:** MiR-375 regulates the effect of YAP1 on the invasion of HeLa cells. (a) Cell invasion in each group after transfection of miR-375 mimic and si-YAP1 (400×); (b) comparison of the number of invaded cells in each group; ^*∗*^*P* < 0.05, compared with the miR-NC group; ^#^*P* < 0.05, compared with the si-NC group.

**Figure 6:** MiR-375 regulates the effect of YAP1 on HeLa cell apoptosis. (a) Apoptosis of each group after transfection of miR-375 mimic and si-YAP1; (b) comparison of apoptosis rate of each group; ^*∗*^*P* < 0.05, compared with the miR-NC group; ^#^*P* < 0.05, compared with the si-NC group.

**Figure 7:** The effect of miR-375-regulating YAP1 on the expression of EMT-related functional proteins. (a) Western blot to detect the expression of *E*-cadherin, *β*-catenin, and vimentin in each group; (b) comparison of the relative content of *E*-cadherin, *β*-catenin, and vimentin in each group; ^*∗*^*P* < 0.05, compared with the miR-NC group; ^#^*P* < 0.05, compared with the si-NC group.

**Table 1:** MiR-375 and U6 PCR primer sequence.

Name	Project	Sequence (5′‒3′)
MiR-375	Forward primer	AGCCGTTTGTTCGTTCGGCT
	Reverse primer	GTGCAGGGTCCGAGGT

U6	Forward primer	CTCGCTTCGGCAGCACA
	Reverse primer	ACGCTTCACGAATTTGCGT

## Data Availability

The data used or analyzed during the study are available from the corresponding author.
